# 64-Slice Spiral Computerized Tomography under Algebraic Reconstruction Algorithm in the Surgical Treatment of Acquired Immune Deficiency Syndrome Complicated with Gastric Cancer

**DOI:** 10.1155/2022/8548760

**Published:** 2022-06-03

**Authors:** Ke Yang, Zheng Chen, Dayong Xu, Fang Peng

**Affiliations:** ^1^Department of Infection Surgery, The First Hospital of Changsha, Changsha 410005, Hunan, China; ^2^Department of General Surgery, The First Hospital of Changsha, Changsha 410005, Hunan, China; ^3^Department of Science and Education, Changsha Center for Disease Control and Prevention, Changsha 410000, Hunan, China

## Abstract

In order to deeply analyze the application of CT images based on artificial intelligence algorithm in clinical treatment of AIDS patients with gastric cancer, and to provide reference for intervention of AIDS patients with gastric cancer, a total of 100 AIDS patients with gastric cancer were included as the research objects. The patients with CD4+ T lymphocyte count less than 200 cells/*µ*L were in the control group (50 cases), whereas those higher than 200 cells/*µ*L were in the experimental group (50 cases). All the patients underwent 64-slice spiral CT scanning. An improved algebraic reconstruction technology (ART) under L0 algorithmic approach (L0-ART) was proposed, and compared with the total variation (TV), filtered back projection (FBP), and weighted total variation (WTV) models. The standard deviation (STD) and average processing time of the L0-ART algorithm were significantly lower than those of the TV, FBP, and WTV algorithms (*P* < 0.05). The operation time of the experimental group was longer than that of the control group; the intraoperative blood loss, the diameter of the surgical wound, the time of first farting, the length of hospital stays, and the incidence of adverse reactions were all greatly lower than those of the control group (*P* < 0.05). Postoperatively, the total adipose tissue (TAT), visceral adipose tissue (VAT), and subcutaneous adipose tissue (SAT) in the abdominal area were higher in the experimental group than those in the control group (*P* < 0.05). In conclusion, the improved L0-ART algorithm proposed in this study had an excellent processing effect on CT images with a clinical promotion value. Patients with CD4+ T lymphocytes over 200 cells/*µ*L had better surgical outcomes and prognosis than those with less than 200 cells/*µ*L.

## 1. Introduction

The ability to resist infection and tumor defense in patients with acquired immune deficiency syndrome (AIDS) decreased due to immunodeficiency. It is very easy to complicate with various tumors, and the probability of suffering from tumors is about 50 times of the normal population [1–3]. The most common tumors in AIDS patients are Kaposi's sarcoma and lymphoma (Burkitt lymphoma, central nervous system lymphoma, diffuse large B-cell lymphoma, etc.), in addition to aggressive cervical cancer, lung cancer, anal cancer, Hodgkin's lymphoma, liver cancer, prostate cancer, and so on [4]. Relevant studies have shown that the number of CD4+ T lymphocytes in patients continues to decrease, and the decline in cellular immune function is the main cause of opportunistic infections and malignant tumors in the body. When the human immunodeficiency virus (HIV) gets into the body, it produces a large number of viruses to invade and destroy T cells. T cells are progressively reduced, the ratio of CD4/CD8 cells is inverted, and cellular immune function is impaired [5–7]. The overall decrease in T lymphocytes shows severe cellular immunodeficiency, creating conditions for rapid growth, metastasis, and secondary infection of tumors, and the probability of opportunistic infections and malignant tumors increases significantly [8, 9]. At present, gastric cancer in AIDS patients cannot be treated with surgery, and the tumor progression can only be controlled by chemotherapy, and analgesic drugs can be given to relieve the pain of patients. However, patients with low immunity may suffer from relatively great side effects [10].

Computed tomography (CT) is to use precisely collimated X-ray beams, gamma rays, ultrasonic waves, etc., together with a highly sensitive detector for the profile scanning of a certain part of the human body one by one, with a short scanning time, clear images, and other characteristics [11, 12]. Nowadays, CT has been widely used in human disease screening, especially for the evaluation of disease progression and chemotherapy efficacy in tumor patients, making it a direct, reliable, and convenient examination method [13]. However, as there are a large number of organs in the human body, the density difference among the organs is small, and the contrast is poor, the obtained original CT images often have a lot of noise and artifacts with a poor quality, which affects the judgment of the radiologist. Thus, the original images need to be enhanced with the help of artificial intelligence algorithms [14–16]. The algebraic reconstruction technology (ART) is to reconstruct the image by solving the system of linear equations. Starting from a hypothetical initial image, it uses a step-by-step approaching method. The theoretical projection value and the actual measured projection value are continuously compared and iteratively updated until the optimal solution is obtained, which was first applied in positron emission CT imaging [17–19]. ART can produce better high-quality images under the condition of low radiation dose, so it was intended to build the ART to segment and reconstruct original CT images, to improve the accuracy of imaging examinations.

In summary, the combination of artificial intelligence algorithms and CT imaging technology is a hot topic in the diagnosis and treatment of diseases currently. But the image reconstruction performance of artificial intelligence algorithms will affect the quality of CT images easily. Therefore, 100 patients with AIDS and gastric cancer who underwent radical gastrectomy were analyzed. Their surgical conditions, postoperative adverse events, and body fat parameters under different immune levels were compared. It was intended to explore the surgical treatment effect and prognosis of AIDS patients with gastric cancer under the ART-based algorithm and CT images.

## 2. Materials and Methods

### 2.1. Research Objects

A total of 100 patients with AIDS complicated with gastric cancer were included as the research objects, who were diagnosed and received radical gastrectomy in hospital from December 20, 2018 to May 20, 2020. This includes 63 males and 37 females, with the age of 39–75 years old. Patients with CD4+ T lymphocyte count less than 200 cells/*µ*L were in the control group (50 cases), and those with CD4+ T lymphocyte count higher than 200 cells/*µ*L were in the experimental group (50 cases). This study had been approved by the ethics committee of the hospital. All the patients and their families were aware, participated in the research voluntarily, and signed the informed consent form before the implementation of the project.

Inclusion criteria were patients had no history of anticancer treatment before surgery; they signed the informed consent voluntarily; and they could offer the complete clinical data.

Exclusion criteria were patients dropped out of the project halfway; they were complicated with other malignant tumors; and they were younger than 20 years old, were complicated with mental diseases, had poor compliance with examinations, or were complicated with metabolic diseases such as diabetes.

### 2.2. CT Scanning Method

A 64-slice dual-source CT scanner was performed. The scanning parameters included tube voltage 120 kV, tube current 200 mA, layer thickness 2.5 mm, layer spacing 2.5 mm, pitch 0.8, and collimator width 0.55 mm. The intravenous injection with 100 mL iopromide (350 mgI/mL) was given via the cubital vein with a syringe, and then the three-phase contrast-enhanced scanning was conducted. The intelligent tracking technology was adopted in the arterial phase. When the abdominal CT value was greater than 150 HU, the scanning started; it was delayed by 20 seconds in the venous phase and delayed by 180 seconds in the delay phase. The original CT images were sent to the workstation, the relative area of interest was outlined, and the abdominal area of total adipose tissue (TAT), visceral adipose tissue (VAT), and subcutaneous adipose tissue (SAT) were calculated.

### 2.3. Improved ART under L0 Algorithmic Approach

The theory of compressed sensing included two parts, one was the observation value obtained by projecting on the observation vector, and the other was to construct the signal by using the ART. First, it was assumed that the length of the signal was *L*, and the sparsity was *M*, then the projection of the signal on the observation vector could be expressed as (1).

(1) $$\begin{array}{c} p_{i}=\langle \lambda ,\varepsilon \rangle ,\;i=1,2,\ldots ,n,\;n<L. \end{array}$$

In the equation, *p*_*i*_ represented the sampling value obtained by compressed sensing with the number of *n*. *ℜ* was the observation base composed of a set of observation vectors (*ϕ*_*i*_)_*i*=1_^*n*^. The key to construct a signal was to find the sparse representation of the signal in a certain variation domain ∀, which could be solved by means of the L0 norm optimization in (2).

(2) $$\begin{array}{c} \min{\left\|\forall \varepsilon \right\|}_{0}\begin{array}{cc} \partial t, & p=\phi \end{array}\varepsilon . \end{array}$$

Later, the image solution with a sparse structure was found through the 0-norm optimization, and then (2) could be updated as (3).

(3) $$\begin{array}{c} \min{\left\|\varepsilon \right\|}_{0}\begin{array}{cc} \partial t, & p=\phi \end{array}\varepsilon . \end{array}$$

To represented the image to be reconstructed, and ‖*ε*‖_0_=∑_*i*∈*℧*_1[|*ε*(*i*)| > 0], *p* represented the measurement data, *ϕ* represented the measurement matrix, and stood for the image space. Equation (3) described a nondeterministic polynomial issue, which was generally solved by the norm. But for extremely under-sampled data, it was unreliable to solve the issue with L2 norm. Thus, the nonconvex issue was transformed into an optimization issue for solving L1, which was expressed as (4).

(4) $$\begin{array}{c} \min{\left\|\varepsilon \right\|}_{1}\begin{array}{cc} \partial t, & p=\phi \end{array}\varepsilon . \end{array}$$

Gk represented that ‖*ε*‖_1_=∑_*i*∈*℧*_|*ε*_1_|. Then the optimal solution was achieved by approaching the L0 norm step by step. The P-norm equation of the vector was set as (5).

(5) $$\begin{array}{c} {\left\|\varepsilon \right\|}_{P}={\sum_{i}\left|\varepsilon_{i}\right|}^{P},\;0\leq P\leq 2. \end{array}$$

When the *P* value was smaller, the closer it was to the L0 norm. A smooth function was constructed as an approximation of the L0 norm, and the 0 norm could be expressed in the form of the limit as (6).

(6) $$\begin{array}{c} {\left\|\varepsilon \right\|}_{0}=\underset{v⟶0}{\lim}{\sum_{i\in ℧}\left|x\left(i\right)\right|}^{P}. \end{array}$$

It could be obtained that the Lv function was the optimal approximation of the L0 norm, then there was a function as (7) that satisfied the above relationship.

(7) $$\begin{array}{c} \underset{\beta ⟶0}{\lim}\sum_{i\in ℧}v\left(\left|x\left(i\right)\right|,\beta \right)=\sum_{i\in ℧}1\left[\left|x\left(i\right)\right|>0\right]. \end{array}$$

In the equation, *β* was the scaling function. When a signal could be constructed by minimizing the L1 norm, it was guaranteed to construct a signal for any *v* satisfying conditions. Equation (3) was then updated as (8).

(8) $$\begin{array}{c} \min v\left(\phi \varepsilon ,\beta \right)\partial t,\;p=\phi \varepsilon . \end{array}$$

By solving (8), the reconstructed image could be obtained, and the energy function of (8) can be expressed as (9).

(9) $$\begin{array}{c} H\left(x,\beta ,\kappa \right)=\sum_{i\in ℧}v\left(\left|\phi x\left(i\right)\right|,\beta \right)+\frac{\kappa {\left\|\forall x-y\right\|}^{2}}{2}. \end{array}$$

Then the Euler–Lagrange equation of (9) was solved to obtain the solution of the reconstructed image, and (10) and (11) were worked out.

(10) $$\begin{array}{c} R\left(x,\beta ,\kappa \right)=\phi^{\prime \prime }\Lambda \left(x\right)\phi x+\kappa \phi^{\prime \prime }\left(\phi x-y\right)=0, \end{array}$$

(11) $$\begin{array}{c} \Lambda \left(x\right)=\frac{v\left(\left|\phi x\right|,\beta \right)}{\left|\phi x\right|}. \end{array}$$

Therefore, the algorithm process of the ART constructed could be expressed as equations (12)–(16).

(12) $$\begin{array}{c} x=\phi^{\prime \prime }\phi g,\;\beta \gg 0, \end{array}$$

(13) $$\begin{array}{c} \text{while}\left[\frac{{\left\|x-x_{o}\right\|}_{2}}{{\left\|x_{o}\right\|}_{2}}\right]\geq \mu_{o}, \end{array}$$

(14) $$\begin{array}{c} \gamma =\frac{x^{\prime \prime }x}{{\left\|x_{o}\right\|}_{2}},\;x_{o}=x,\beta =\beta \gamma , \end{array}$$

(15) $$\begin{array}{c} \text{while}\left[\frac{{\left\|x-x_{\text{in}}\right\|}_{2}}{{\left\|x_{\text{in}}\right\|}_{2}}\right]\geq \mu_{\text{in}}, \end{array}$$

(16) $$\begin{array}{c} x^{t+1}=-R\left(x^{t},\kappa \right). \end{array}$$

In the equations, *x*_*o*_ represented the outer iteration, whereas *x*_*in*_ represented the inner iteration. The inner iteration iterated all the data, and a simple iterative operation was carried out under the condition of setting a parameter. The outer layer was gradually approaching the L0 norm as the parameter decreased. When the outer iteration result was not different from the original image, the reconstructed image could be obtained. The improved ART under L0 algorithmic approach proposed here was set as L0-ART.

### 2.4. Algorithm Simulation Experiment

The total variation (TV) model [20], filtered back projection (FBP) algorithm [21], and weighted total variation (WTV) model [22] were introduced and were compared with the L0-ART algorithm.

The standard deviation (STD) of the reconstructed images [23] and the average reconstruction time were taken as evaluation indicators. STD could be expressed as (17), together with (18) and (19).

(17) $$\begin{array}{c} \text{STD}=\sqrt{\frac{\sum_{x=1}\sum_{y=1}{\left[f\left(x,y\right)-\bar{f}\right]}^{2}}{D^{2}}}, \end{array}$$

(18) $$\begin{array}{c} f\left(x,y\right)=a\left(x,y\right)-a_{0}\left(x,y\right), \end{array}$$

(19) $$\begin{array}{c} \bar{f}=\sum_{x=1}^{d}\sum_{y=1}^{d}f\left(x,y\right). \end{array}$$

In the equations, *a*(*x*, *y*) represented the reconstructed image, whereas *a*_0_(*x*, *y*) represented the original image.

### 2.5. Observation Indicators

The basic information of patients, including gender, age, tumor diameter, tumor stage, tumor grade, body mass index (BMI), preoperative TAT, VAT, and SAT, were recorded. The surgical conditions of the patients (operation time, intraoperative blood loss, surgical wound diameter, time of first farting, and length of hospital stay) were also recorded. The patients were followed up after surgery, and adverse events (gastrointestinal dysfunction, wound infection, anastomotic leakage, pulmonary infection, and pleural effusion) were recorded as well.

### 2.6. Statistical Processing

SPSS19.0 was used for data processing. Measurement data were expressed as mean ± standard deviation $a\left(\bar{x}\pm s\right)$, and enumeration data were expressed as percentage (%). Pairwise comparisons were made using a one-way analysis of variance. The difference was statistically significant at *P* < 0.05.

## 3. Results

### 3.1. Simulation Results of Different Algorithms

As shown in Figure 1, the STD and average processing time of the L0-ART algorithm were significantly lower than those of the TV model, FBP algorithm, and WTV model, with statistically significant differences (*P* < 0.05).  Figure 2 displayed the reconstructed images of the four algorithms. It could be observed that compared with the original CT image, the reconstructed images were significantly improved in terms of sharpness and contrast. The L0-ART algorithm reconstructed the image with the least noise and artifacts, having the highest overall quality.

### 3.2. Imaging Data of Some Patients

The imaging data of a 65-year-old male patient were shown in Figure 3. The physical examination suggested nothing special. The gastroscopy showed that the nature of the pyloric ulcer was to be investigated, and there was chronic superficial erosive gastritis, local mucosal atrophy of the gastric fundus, and mucosal bulge of the gastric body. Abdominal CT examination showed that the gastric wall of pylorus was thickened, and invasive gastric cancer was not ruled out.

The imaging data of a 70-year-old female patient was shown in Figure 4. The physical examination revealed no abnormality in cardiopulmonary auscultation, and the abdomen was flat. The patient got mild epigastric pressing pain, with no rebound tenderness and muscle tension. No gastrointestinal pattern or peristaltic wave was discovered, with normal bowel sounds and negative moving dullness. It was shown with poorly differentiated adenocarcinoma through gastroscopy. CT scanning revealed a thickening of the gastric wall in the corners of the stomach.

### 3.3. Comparison of the Basic Data between the Two Groups of Patients

As shown in Figure 5, the gender ratio, average age, BMI, tumor staging (phase I, II, III, and IV), and pathogenic site (cardiac part, lesser curvature, and gastric antrum) of patients were compared between the experimental group and the control group. The differences in the pairwise comparisons were not statistically significant (*P* < 0.05).

### 3.4. Comparison of Surgical Conditions between the Two Groups of Patients

As shown in Figure 6, the operation time of the patients in the experimental group was significantly longer than that in the control group, with the difference statistically significant (*P* < 0.05). The intraoperative blood loss, surgical wound diameter, time of first farting after surgery, and the length of hospital stay of patients in the experimental group were all significantly lower than those of the control group, indicating the statistically significant differences (*P* < 0.05).

### 3.5. Postoperative Adverse Events of Patients in the Two Groups

As shown in Figure 7, there were two cases complicated with gastrointestinal dysfunction, three cases with wound infection, two cases with anastomotic leakage, four cases with pulmonary infection, and one case with pleural effusion after surgery in the control group. For patients in the experimental group after surgery, there were one, one, zero, two, and zero cases complicated with gastrointestinal dysfunction, wound infection, anastomotic leakage, pulmonary infection, and pleural effusion, respectively. The incidence of postoperative adverse events in the experimental group (8%) was significantly lower than that in the control group (24%), and the difference was statistically significant (*P* < 0.05).

### 3.6. Comparison of Body Fat Parameters of Patients before and after Surgery between the Two Groups

As shown in Figure 8, the body fat parameters TAT, VAT, and SAT after surgery were significantly lower than those before surgery in both the experimental group and the control group, with statistically significant differences (*P* < 0.05). No statistically significant difference was found in the preoperative TAT, VAT, and SAT between the experimental group and the control group (*P* > 0.05). The postoperative TAT, VAT, and SAT in the experimental group were significantly higher than those in the control group, and the differences were statistically significant (*P* < 0.05).

## 4. Discussion

HIV has a strong attack on the human immune cells dominated by CD4+ T lymphocytes, gradually leading to the damage and loss of the human immune system, and eventually resulting in AIDS-related malignant tumors. The differential diagnosis of different AIDS-related malignancies is very important for the prognosis of patients with surgical treatment [24]. Given that the original image will be affected by objective conditions such as the doctor's operation technique and the patient's posture, the improved L0-ART algorithm was put forward. Compared with the TV model, the FBP algorithm, and the WTV model in the simulation experiment, it was suggested from the results that the STD and average processing time of the L0-ART algorithm were significantly lower than those of the TV model, the FBP algorithm, and the WTV model (*P* < 0.05). The smaller the STD, the better the reconstructed image. This result proved that compared with the traditional algorithms, the quality of reconstructed CT image processed by the L0-ART algorithm was better, and the reconstruction took less time. It was beneficial to improve the accuracy and efficiency of diagnosis and to assist radiologists in objective assessment [25]. The reconstructed image by the four algorithms was further compared, from which it was observed that the reconstructed images had been significantly improved in terms of clarity and contrast compared with the original CT image. The L0-ART algorithm reconstructed the image with the least noise and artifacts, and the overall quality was also the highest. This was consistent with the above results of quantitative indicators, confirming the superiority of the L0-ART algorithm once again.

A total of 100 patients with AIDS complicated with gastric cancer and underwent radical gastrectomy were selected as the research objects. The patients with CD4+ T lymphocyte count less than 200 cells/*µ*L were included as the control group, 50 cases. Those with CD4+ T lymphocyte count higher than 200 cells/*µ*L were included in the experimental group, 50 cases as well. First, the basic data of patients were compared between the two groups, and it was known that there was no statistically significant difference of the pairwise comparisons in the gender ratio, average age, BMI, tumor staging (phase I, II, III, and IV), as well as pathogenic site (cardiac part, lesser curvature, and gastric antrum; *P* < 0.05). Such a result provided feasibility for follow-up research. The surgical conditions of patients in both the groups were compared, and found that the operation time of the experimental group was significantly longer than that of the control group, while the intraoperative blood loss, surgical wound diameter, time to first farting, and length of hospital stay were significantly lower than those of the control group (*P* < 0.05). This was similar to the findings of Aliaga Ramos et al. [26], indicating that there were significant differences in the results of radical gastrectomy for patients with different immune levels. The surgical conditions of the patients with CD4+ T lymphocytes higher than 200 cells/*µ*L were better than those below 200 cells/*µ*L. The incidence of postoperative adverse events in the experimental group (8%) was significantly lower than that in the control group (24%) with a difference of statistical significance (*P* < 0.05), which indicated that radical gastrectomy had different effects on the prognosis of AIDS patients complicated with gastric cancer with different immune levels. The surgical prognosis of patients with more than 200 cells/*µ*L CD4+ T lymphocyte count was better than those with less than 200 cells/*µ*L. In addition, the body fat parameters of the patients before and after surgery were also compared, and it was found that the body fat parameters TAT, VAT, and SAT after surgery were significantly lower than those before surgery with statistically significant differences (*P* < 0.05), suggesting that the changes in body composition of patients were obvious after surgery, especially the fat content decreased significantly. The postoperative body fat parameters TAT, VAT, and SAT in the experimental group were significantly higher than those in the control group with the differences of statistical significance (*P* < 0.05). The decreased fat content of patients might be related to inflammatory response, postoperative fasting, low food intake, and increased energy consumption [27]. Patients with higher than 200 cells/*µ*L CD4+ T lymphocyte counts got better surgical conditions and prognosis, as the postoperative fasting time and food intake were decreased, inflammatory responses were reduced, and fat content levels were improved.

## 5. Conclusion

The improved L0-ART algorithm was proposed at first on the grounds of the algorithmic approach of the L0 algorithm. The simulation experiment was carried out to compare the proposed algorithm with the TV model, the FBP algorithm, and the WTV model. A total of 100 AIDS patients complicated with gastric cancer and who received radical gastrectomy were selected as the research objects. There were 50 cases in the control group, as the patients had CD4+ T lymphocytes less than 200 cells/*µ*L and 50 cases in the experimental group whose CD4+ T lymphocytes were higher than 200 cells/*µ*L. Compared with the traditional algorithm, the L0-ART algorithm produced the reconstructed CT images with better quality and less time. It was conducive to improving the diagnostic accuracy and efficiency, and assisting radiologists in objective evaluation. For patients with different immune levels, radical gastrectomy had significantly different surgical effect and prognosis on patients. The surgical effect and prognosis of patients with CD4+ T lymphocyte count more than 200 cells/*µ*L were better than those of patients with less than 200 cells/*µ*L. However, there are still some deficiencies in this research. The sample size of the patients included was small and the sample source was single, thus there might be sampling errors, having some impact on the data results. The time of follow-up was short, and more prognosis might be missed. The sample size would be increased, and more follow-up investigations would be made later. In summary, the results provided a data reference for the application of artificial intelligence algorithms combined with CT influence in clinical surgical treatment.

## Figures and Tables

**Figure 1:** Comparison of the performance indicators of four algorithms in the reconstruction of images. (a) STD; (b) processing time. ^*∗*^Compared with the data of the L0-ART algorithm, *P* < 0.05.

**Figure 2:** Results of reconstructed CT images by four algorithms. (a) The original image; (b, c, d, and e) the reconstructed images processed by the TV model, FBP algorithm, WTV model, and L0-ART algorithm, respectively.

**Figure 3:** Imaging data of a 65-year-old man who visited the doctor because of epigastric discomfort for 2 weeks. (a) and (b) were the results of gastroscopy, while (c) and (d) were CT images.

**Figure 4:** Imaging data of a 70-year-old woman with persistent pain and discomfort in the upper abdomen for 3 weeks before visiting the hospital, and with the worsened pain in the past 1 week. (a) and (b) were the results of gastroscopy, while (c) and (d) were CT images.

**Figure 5:** Comparison of basic data of patients between the two groups. (a), (b), (c), and (d) show the comparison of gender, average age and BMI, tumor staging, and pathogenic site, respectively.

**Figure 6:** Comparison of the surgical conditions of the two groups. (a) The comparison of the operation time and intraoperative blood loss; (b) the diameter of the surgical wound; (c) the time of first farting and the length of hospital stay. ^*∗*^Compared with those of the experimental group, *P* < 0.05.

**Figure 7:** Postoperative adverse events in the two groups. (a) The number of cases of gastrointestinal dysfunction, wound infection, anastomotic leakage, pulmonary infection, and pleural effusion; (b) the incidence of adverse events. ^*∗*^Compared with that of the experimental group, *P* < 0.05.

**Figure 8:** Comparison of body fat parameters before and after surgery in the two groups. (a), (b), and (c) represent the comparison of TAT, VAT, and SAT, respectively. ^*∗*^Compared with the experimental group, *P* < 0.05.

## Data Availability

The data used to support the findings of this study are available from the corresponding author upon request.
